The article "Optimization Method of an Antibreast Cancer Drug Candidate Based on Machine Learning" was published in 2022. Journal: Comput Math Methods Med.

# Optimization Method of an Antibreast Cancer Drug Candidate Based on Machine Learning

**DOI:** 10.1155/2022/4133663

**Published:** 2022-09-05

**Authors:** Zhibai Huang, Shengji Jiang, Weiqiang Xiao

**Affiliations:** East China Institute of Computing Technology, Shanghai, China

## Abstract

Breast cancer is a common but serious and even lethal disease. Fortunately, compared with other cancers, breast cancer treatments currently are relatively well developed. The use of specific drugs is typically essential in the majority of breast cancer treatment strategies. Given the aforementioned factors, it is important to continue researching effective antibreast cancer drug design. Machine learning-based computer-aided drug design is currently a common practice in both drug industries and academic institutes. According to the characteristics of breast cancer, we selected multiple candidate compounds; based on the corresponding molecular descriptors, biological activities, and pharmacokinetic properties, a dataset of inhibition potency and pharmacokinetic properties paired with multiple features of compounds was constructed. On this basis, the random forest method was utilized to choose greater-influenced feature embeddings; thus, 224 main operating variables were selected for further analysis; we then employed the efficient MobileNetV3 deep neural network as the backbone to establish the prediction models for the inhibition potency and pharmacokinetic properties of the compounds. After data preprocessing, the weights are obtained by training on the refined dataset. Finally, we define an optimization problem to discover compounds with the best properties. The problem is solved using the genetic algorithm with the acquired prediction model, and the solution value for the corresponding operating variables with the best clinical properties in theory is then obtained. Analysis demonstrates that our approach could be used to aid the screening process of antibreast cancer drug candidates.

## 1. Introduction

Breast cancer currently ranks among the most prevalent cancers worldwide [1] and has a high fatality rate. Estrogen receptors are connected with the development of breast cancer [2, 3]. Given that the estrogen receptor *α* subtype (estrogen receptor alpha (ER*α*)) is present in roughly 70% of breast cancer cells [4], it has been widely considered in the diagnosis of breast cancer [2]. Studies on mice with ER*α* gene modifications have demonstrated that ER*α* does, in fact, play a crucial role in the development of the uterus and mammary glands [4, 5]. Consequently, as ER*α* is considered a key target for the treatment of breast cancer, substances that can suppress ER*α* activity might be proper candidates for use as therapeutics [2].

The article "Optimization Method of an Antibreast Cancer Drug Candidate Based on Machine Learning" was published in 2022. Journal: Comput Math Methods Med.

For a long time, the gold standard for the endocrine treatment of several breast cancer types was tamoxifen [6], a common drug with estrogen-like actions. Since tamoxifen was found to be effective in treating breast cancer, numerous studies have been conducted to highlight the significance of hormone therapy for the disease [7, 8]. In addition to hormone therapy, other medicines for breast cancer include chemotherapy and immunological therapy [9]. As the leading drugs for the aforementioned therapies, cyclophosphamide, docetaxel, pertuzumab, and trastuzumab are currently commonly used to treat breast cancer [10–13].

Building an inhibitory potency prediction model can be used to screen candidate compounds during the conventional drug design process to save time and money [14]. The precise procedure is as follows: first, for a biological target associated with a disease, gather data on a number of compounds that affect the target and their biological activity. Next, build a quantitative structure-activity relationship (QSAR) model of candidates using a number of molecular descriptors as independent variables and the biological activity value of the compound as the dependent variable. Finally, the model is employed to forecast how a molecule might seem when having sufficient biological activity or to direct the structural improvement of already existing compounds [15].

In addition to having significant biological activity, a chemical should also have appropriate pharmacokinetic and safety qualities in the human body to be employed as a new medicine. Similar to that, it can be evaluated using an established QSAR model [16]. There are numerous ways to create prediction models at the time, whereas methods based on artificial neural networks have received more attention from academic communities than other alternatives [15, 17, 18]. Computer-aided drug design techniques have been applied extensively in many aspects of drug design after years of development [19, 20]. Deep neural networks have been extensively used since the dawn of the big data age, and numerous research in drug design have been conducted [21, 22]. A few researchers have attempted to use the effective convolutional neural network MobileNetV3 [23] in the field of medicine [24, 25].

In this research, based on the current knowledge, we created a dataset of potential antibreast cancer drug candidates, and then, we refined the dataset by applying the random forest algorithm. We explore adopting MobileNetV3 to create a QSAR model on the refined dataset to construct the qualitative model of pharmacokinetic performance and the quantitative prediction model of inhibitory potency. Finally, a problem for optimizing the attributes of the chemical is created based on the model that was obtained and the genetic algorithm is utilized to solve the problem.

The article "Optimization Method of an Antibreast Cancer Drug Candidate Based on Machine Learning" was published in 2022. Journal: Comput Math Methods Med.

## 2. Dataset Construction and Preprocessing

### 2.1. Dataset Construction

According to prior knowledge and experience, we selected a total of 1974 compounds, calculated the corresponding 2-dimensional and 3-dimensional molecular descriptors by computing software [26], and subsequently marked their biological activity values and ADMET properties to complete the construction of the dataset. We choose IC50, pIC50 as the index for biological activity, Caco-2 for A (absorption), CYP3A4 for D (distribution), hERG for M (metabolism), HOB for E (excretion), and MN for T (toxicity). Specifically, Caco-2 is the permeability of small intestinal epithelial cells, which can measure the ability of the compound to be absorbed by the human body. CYP3A4 is the cytochrome P450 enzyme 3A4 isoform, which is the main metabolic enzyme in the human body, which can measure the compound. hERG is the cardiac safety evaluation of the compound, which can measure the cardiotoxicity of the compound. HOB is the oral bioavailability of the human body, which can measure the proportion of the drug absorbed into the human blood circulation after entering the human body. MN is the micronucleus test and is a method to detect whether a compound is genotoxic.

Based on the dataset (including 1974 compound samples, each with 1361 molecular descriptor variables, e.g., electrotopological state atom type descriptor, ring count descriptor, WHIM descriptor etc., 2 biological activity data, and 5 ADMET property data), we then built a quantitative prediction model for compound biological activity and a categorical prediction model for ADMET properties.

### 2.2. Data Preprocessing

#### 2.2.1. Data Cleaning

Due to some problems in the collected raw data, to ensure the data analysis quality, the raw data should be cleaned in a certain level. The overall data processing method is as follows:

1. There is dimensionless normalization of molecular descriptor data in all samples
2. For data columns with most of the data being 0, delete them directly
3. Only the pIC50 array was selected as the biological activity label

Considering the large difference in raw values between different molecular descriptors, to improve the model accuracy, we first use the min-max normalization method [27] to perform dimensionless normalization on the molecular descriptor data.

On this basis, we double check the normalized samples and delete most of the data columns with 0 values (dimensionless normalized molecular descriptors) to reduce data redundancy. Make datasets more compact and efficient without losing too much information. By excluding some factors with low impact on biological activity in advance, the convergence speed of subsequent selection of main features should be accelerated.

The article "Optimization Method of an Antibreast Cancer Drug Candidate Based on Machine Learning" was published in 2022. Journal: Comput Math Methods Med.

Finally, we chose pIC50 as the only numerical annotation for biological activity. Since the pIC50 value is distributed in the [0, 10] interval, it is more friendly to the deep network model. Considering that the IC50 and pIC50 can be equivalently transformed through numerical calculation, dropping the IC50 label should not ignore valuable information. Only pIC50 is selected as the biological activity numerical labeling instead of the IC50 and pIC50 binary label group; we believe that the sole existence of pIC50 should make the dataset more “compact,” thus leading to a more efficient and accurate prediction model.

#### 2.2.2. Selecting Main Features

Considering the large number of data columns in the dataset, it is necessary to further compress the number of data columns; we chose to use the random forest algorithm [28] to select features to further compress the dataset. The importance of each feature can be obtained by performing certain operations on the result of the sample classification. The smaller the result is, the smaller impact that this feature affects the prediction result. According to the variable contribution ranking obtained by random forest algorithm, we select a total of 224 data columns (which are processed molecular descriptors) in order of contribution, as shown in Figure 1.

Among them, XlogP is the lipid-water partition coefficient, which reflects the absorption effect of molecules through the cell membrane. TopoPSA is the topological polar surface area, reflecting factors such as molecular size and solubility. From the statistical results of the categories to which each variable belongs, it can be seen that the extracted variables include a certain level of comprehensive types of compound fingerprints. The variance is relatively minimal, which suggests that the extracted variables place a balanced emphasis on each category, according to the distribution of the number of variables contained in each category. The final selected normalized molecular descriptors are shown in Table 1. After the compressing process, we have done all data preprocessing for the deep neural network.

## 3. Compound Property Prediction Model

### 3.1. Quantitative Prediction Model for Biological Activity

#### 3.1.1. Model Design

Artificial neural networks are currently employed and widely applied in the field of computer-aided drug design. The most often used neural network is the BP (back propagation) neural network, a multivariate feedforward neural network trained via error back propagation. Deep neural networks, a version of BP neural networks, have drawn considerable attention in many fields of academia and industry. Convolutional neural networks among them have significant advantages in performance and are especially well liked in the field of computer vision. However, it is important to keep in mind that the majority of the current popular convolutional neural networks have complex structures, thus containing a lot of parameters, combined with the neural network's data-hungry nature making model training very challenging. Special consideration should be given when training these networks on relatively small-amount biological activity datasets.

The article "Optimization Method of an Antibreast Cancer Drug Candidate Based on Machine Learning" was published in 2022. Journal: Comput Math Methods Med.

On the other hand, it is crucial to properly design the number of neurons in the hidden layer during the whole network construction process. The workload required to make the network function will significantly arise if the hidden layer contains too many neurons, which can quickly result in an undesired overfitting issue. Conversely, if the hidden layer contains too few neurons, which will also negatively affect the network's quality, thus resulting in poor prediction accuracy. The total number of neurons in a neural network's hidden layer is directly correlated with the difficulty of the task, the number of neurons in the input and output layers, and the expected bias settings of those neurons.

Considering the mentioned problems, we chose the MobileNetV3 deep convolutional neural network as the backbone to construct a quantitative prediction model for the biological activity of compounds. As one of the representatives of lightweight models, compared to the classic convolutional network VGG16 [29], MobileNetV3 greatly reduces the number of parameters but is more efficient and easier to train while ensuring similar performance. The schematic diagram of the network structure that we use is shown in Figure 2.

#### 3.1.2. Model Training

We first divide the 1974 group of data in the dataset into training set data (around 80% in amount), test set data (around 15% in amount), and validation set (around 5% in amount) according to the proportions of 80%, 15%, and 5%, respectively. After the division is completed, 224 main variables in the dataset and pIC50 annotations were constructed as a pair; then, randomly sample 10 data pairs as a batch for model input.

As an important part of model optimization, the loss function needs to be carefully considered. Considering that the quantitative prediction problem can be summarized as a regression problem, we choose MSELoss (mean square error loss), the most commonly used one in the regression task, as the loss function.

The article "Optimization Method of an Antibreast Cancer Drug Candidate Based on Machine Learning" was published in 2022. Journal: Comput Math Methods Med.

Deep learning tasks will produce varying results depending on the optimizers used. We first identified the SGD (stochastic gradient descent) [30] and Adam optimizer (adaptive moment estimation optimizer) [31] as alternatives based on the properties of the MobileNetV3 network itself and the properties of the dataset; we then compared the performance in the experimental training, and Adam was ultimately selected as the optimizer.

Finally, considering the nature of the Adam optimizer itself, we adopt the cosine annealing strategy [32] to update the learning rate to optimize the performance of the model as much as possible. In selecting the most suitable upper limit of the hyperparameter learning rate and the number of epochs, we also performed experimental training on the actual training set. Ultimately, we came to the conclusion that the upper limit of the learning rate is 0.0001 and the number of epochs is 100.

### 3.2. Qualitative Prediction Model for ADMET Properties

To simplify the problem, we trained the models separately for the five properties in ADMET. To further simplify the problem, we believe that each property has only two possibilities of “yes” or “no,” which can be expressed by the values 0 and 1. In this way, the problem can be classified as a binary classification problem; then, we can reuse the divided dataset given in Section 3.1.2 and merely change the data label to pharmacokinetic properties.

Since the input data share a certain level of similarity, we still employ the MobileNetV3 structure as the backbone; therefore the desired model structure is essentially identical to the structure described in Figure 2. The only needed minor change is to adjust the output neuron of the bottom fully connected layer and add an extra sigmoid activation function; other designs shall not be repeated here.

To adapt to the binary classification problem, the model training method also needs to be adjusted. We changed the loss function to BCELoss (binary cross entropy loss), while the optimizer, learning rate adjustment strategy, and hyperparameter setup remain unchanged. The prediction accuracy is obtained based on the comparison between the predicted outputs and the real labels.

During the training process based on experiments on real datasets, the issue of data imbalance has been found. To prevent the trained model from being biased due to data imbalance, we redundantly expand the data, that is, expanding the samples of a relatively small number to be roughly equivalent to the other categories.

### 3.3. Optimization Model for Clinical Properties Based on Specific Features

#### 3.3.1. Definition of Optimization Problem

We now define an optimization problem using these six prediction models that were trained in earlier sections, looking for the ideal circumstances for the 224 variable values that were chosen. Note that we assume that any “acceptable” compound must perform “well” at least three of the given ADMET properties; then, the problem could be defined as follows:

**Definition 1 .**

The article "Optimization Method of an Antibreast Cancer Drug Candidate Based on Machine Learning" was published in 2022. Journal: Comput Math Methods Med.

Given the selected molecular descriptor, what value of the molecular descriptor satisfied can make the compound have better biological activity for inhibiting ER*α*, meanwhile having better ADMET properties (at least three or better).

#### 3.3.2. Optimization Problem Modeling

First, determine the decision variables; we follow the selected results in the previous section; consider the selected 224 molecular descriptors as decision variables, denoted as follows:

(1) $$\begin{array}{c} X=\left\{x_{1},x_{2},x_{3},\cdots ,x_{224}\right\}. \end{array}$$

Now, determine the objective function. After analyzing the problem, we can find that the problem essentially is as follows: based on the given prediction models, under the premise that at least three properties of the given five ADMET properties are “good,” by changing the value of selected features, the clinical properties (both inhibition potency and pharmacokinetic performance) are optimized to guide the production process. The biological activity of the compound is altered by the chosen feature's value; it is worth noting that this process will also alter the compounds' ADMET properties. Therefore, the relations between each model should not be ignored. By applying the prediction models to the input samples, the predicted value of ADMET properties of each sample can be obtained. Following the idea in Section 3.2, we take all the values representing good properties as 1 and the values of bad properties as 0; then, we get an optimization limit that the pharmacokinetic point (the sum of ADMET property marks) has a maximum value of 5. According to Definition 1, the ADMET marks of an “acceptable” compound should not be less than 3; then, the modified output function of the qualitative prediction model is derived, denoted original output as *ϕ*(*X*); then, denote our desired function as *Φ*(*X*), defined as follows:

(2) $$\begin{array}{c} \Phi \left(X\right)=\left\{\begin{array}{c} 0,\;0\leq \underset{\text{ADMETproperties}}{\sum }\phi \left(X\right)<3,\\ \underset{\text{ADMETproperties}}{\sum }\phi \left(X\right),\;3\leq \underset{\text{ADMETproperties}}{\sum }\phi \left(X\right)\leq 5. \end{array}\right. \end{array}$$

In addition to the ADMET properties, we need to consider the pIC50 value of the compound as well. The goal of this output function is to obtain the highest activity value under the premise of satisfying “acceptable” ADMET properties; combined with the definition of pIC50, the modified quantitative prediction model output function is given. We denoted it as Ψ(*X*) and the original one as *ψ*(*X*), define as follows:

(3) $$\begin{array}{c} \Psi \left(X\right)=\left\{\begin{array}{c} 0,\;10<\psi \left(X\right),\\ 0,\;\psi \left(X\right)<0,\\ \psi \left(X\right),\;0\leq \psi \left(X\right)\leq 10. \end{array}\right. \end{array}$$

Intuitively, the optimization problem should be a multiobjective nonlinear programming problem. To simplify the solution process, we transform it into a single-objective nonlinear programming problem to solve. Considering the optimization problem, it is desired that the compound's ADMET properties are as good as possible and the biological activity is as high as possible, that is, to find a set of selected feature values *X*_0_ to maximize the sum of *Φ*(*X*_0_) and Ψ(*X*_0_). In this way, we are able to extract the objective function of the optimization problem, which is defined as follows:

(4) $$\begin{array}{c} F\left(X\right)=\Psi \left(X\right)+\Phi \left(X\right). \end{array}$$

Finally, determine the constraints: for this optimization problem, since the proposed 224 decision variables (dimensionless normalized molecular descriptors) have a certain range of actual values, there is constraint 1 as follows:

(5) $$\begin{array}{c} 0\leq x_{i}\leq 1,\;i=1,2,3,\cdots ,224. \end{array}$$

Now, take into account the biological activity limitation. Considering the predicted pIC50 value, according to the definition of pIC50, it can be seen that there is a constraint on the value of *ψ*(*X*) and we hope that the optimized biological activity value is not lower than the maximum value in the dataset for building the prediction model, so there is a constraint 2 as follows:

(6) $$\begin{array}{c} 10\geq \text{pIC}50_{\text{t}\arg\text{et}}\geq \text{pIC}50_{\text{source}}\geq 0. \end{array}$$

Combine constraints with the target function; in summary, the problem can be defined as follows:

(7) $$\begin{array}{c} \begin{array}{c} \text{Max }F\left(X\right)\\ \text{s}.\text{t}.\left\{\begin{array}{c} 0\leq x_{i}\leq 1,\;i=1,2,3,\cdots ,224,\\ 10\geq \text{pIC}50_{\text{target}}\geq \text{pIC}50_{\text{source}}\geq 0. \end{array}\right. \end{array} \end{array}$$

The article "Optimization Method of an Antibreast Cancer Drug Candidate Based on Machine Learning" was published in 2022. Journal: Comput Math Methods Med.

#### 3.3.3. Optimization Problem Solving

We now address the optimization problem raised in Section 3.3.2. It can be said that the optimization problem is a single-objective nonlinear optimization problem given the complicated link between molecular descriptors and biological activity. Intelligent optimization algorithms, such the genetic algorithm [33], ant colony algorithm [34], and particle swarm optimization [35], can be used to solve this type of problem's model to acquire the optimal set of variables. We employ the genetic algorithm to address the optimization problem since it can frequently produce better optimization results more quickly than some traditional optimization methods when solving complex combinatorial optimization problems.  Figure 3 depicts a typical genetic algorithm optimization procedure.

The primary chromosomes of some members of the population are first constructed by performing binary coding on the sample operating variable's initial value, and the chromosomes of the remaining individuals are randomly generated within the value range of the operating variable. To determine the fitness of each chromosome in the population and to calculate the corresponding selection probability matrix, the binary-coded chromosomes are first decoded to the actual values of the altered variables before being input into the ADMET property prediction model and the biological activity prediction model. Chromosomes with higher fitness are more likely to be selected during evolution. Roulette selection is used in the selection strategy. Chromosomes interact with one another and mutate to create new chromosomes. Finally, if a combination of operational variables satisfies all requirements for biological activity and pharmacokinetic features, record the combination and optimize the following sample; if not, keep iterating until the ideal operating circumstances are discovered.

We built the solver in Python language to lessen the implementation's complexity. When using a genetic algorithm, simulating more complex “populations” takes longer and takes more effort. After simulation training and testing, we find the proper parameters for the solver. We randomly created the initial population and fixed the number to 2000, taking into account the difficulty of solving and the accuracy requirements. The number of iterations is limited to 500. As for the chromosomes, the number is set to 224, the length of each chromosome is set to 20 bits, the crossover rate is set to 0.6, and the mutation rate is set to 0.1. Record the value of the operand variable that maximizes the objective function, and return it.

## 4. Experimental Results and Discussions

### 4.1. Analysis of the Biological Activity Prediction Model

Once the network has been trained, the prediction can be made by simply feeding the network the values of the main variables. The validation set was imported into the model after establishing the quantitative neural network-based prediction model of biological activity. The predicted outcomes were compared with their real labels, which are displayed in Table 2.

The article "Optimization Method of an Antibreast Cancer Drug Candidate Based on Machine Learning" was published in 2022. Journal: Comput Math Methods Med.

The change curve of the predicted value and its corresponding actual value are similar in Figure 4, which shows that the model has a decent prediction result and is able to accurately reflect the biological activity in theory. The mean square error of the model is 1.572, which is within the acceptable range when choosing MSE to measure the prediction accuracy.

### 4.2. Analysis of the ADMET Property Prediction Model

Compare the predicted results with the actual results by importing the validation set into the trained ADMET property prediction model. The following table display the findings (Table 3).

The verification results for all five attributes are acceptable as considering the aforementioned tables, while the results for HOB are a little inferior. Nevertheless, the accuracy rate is still quite good. The prediction accuracy of HOB is the lowest result in terms of these five attributes, and this fact might be caused by data imbalance, since the neural network-based models tend to develop a preference on biased data. However, our model's average prediction accuracy is close to 85%, which is quite a satisfactory performance.

### 4.3. Analysis of the Clinical Property Optimizing Model

By resolving the optimization problem, the optimal fitness value of 13 is discovered and the relevant actual values for the molecular descriptors are resolved.  Table 4 shows the values of the first 224 molecular descriptors in detail.

It can be found that due to the inconsistency of the definitions among the descriptors, the value difference is relatively large but it seems to not affect the results at last. Consider Figure 5, since the dataset that we created has a maximum fitness value of 12.86 while an optimal fitness value of 13 that could be attained by solving the problem; this fact proves that, by applying our method to existing chemical data, it might be possible to find a candidate which has better properties.

## 5. Conclusion

Breast cancer, as a common and influential disease, requires the development of new drugs to continuously improve the treatment methods. How to efficiently select possible drug candidates to reduce the cost of drug development has a certain research value. In our work, we consider the use of machine learning methods to assist in the selection of compounds. We first used the known knowledge and computer compound molecular descriptor calculation software to construct a dataset and then used the random forest algorithm to screen the features and simplify the dataset; then, based on the MobileNetV3 structural deep convolutional network, the biological activity and pharmacokinetics were constructed.

The article "Optimization Method of an Antibreast Cancer Drug Candidate Based on Machine Learning" was published in 2022. Journal: Comput Math Methods Med.

The invention of novel medications is necessary for the ongoing development of effective treatments for breast cancer, a common and notable disease. There may be some research value in how to effectively choose potential medication candidates to lower the cost of drug development. In our study, we take into account the application of machine learning techniques to aid in compound selection. First, a dataset was created by combining already known inhibition potency knowledge and the compound molecular descriptors generated by modern calculation software. Next, features were screened out and the dataset was made simpler using the random forest algorithm. Finally, the MobileNetV3 structural deep convolutional network was introduced to construct the biological activity and pharmacokinetics. A genetic algorithm solver is utilized to solve an optimization problem based on the obtained prediction model to predict the best value for the chosen molecular descriptors. The analysis from the perspective of the entire drug design process, rather than constructing or modifying each child model, reflects the proposed model's innovation and applicability the most. The internal connection and progressive relationship of each model are emphasized in many places throughout this paper. We believe that our four-step method of influencing variable screening, biological activity prediction modeling, pharmacokinetic properties modeling, and clinical property optimization can successfully model and optimize the properties of drugs through various machine learning technologies and serve as a useful guide for drug manufacturers. According to the aforementioned analysis, our method not only offers a significant practical industrial application value but also some academic innovation and research value.

In the future, our research direction will mainly focus on giving weight to the properties of ADMET. For example, for the properties of hERG, we do not want the drug to be highly toxic to the human body, so for toxic compounds, we will appropriately reduce its evaluation, that is, the calculated adaptation value. Other properties are the same, and we expect to obtain antibreast cancer drugs with better efficacy and less harm to the human body through this method.

## Figures and Tables

**Figure 1:** Visualization of the top 15 variables of contribution.

**Figure 2:** The schematic diagram for the model built.

**Figure 3:** Flowchart of genetic algorithm.

**Figure 4:** Performance of the quantitative prediction model.

The article "Optimization Method of an Antibreast Cancer Drug Candidate Based on Machine Learning" was published in 2022. Journal: Comput Math Methods Med.

**Figure 5:** The figure of best fitness trending.

**Table 1:** The contribution of the top 224 important molecular descriptors (from low to high).

Descriptor	Importance
Smax11	0.00065
MATSp7	0.00065
CIC4	0.000652
MDEC-14	0.000656
S17	0.000659
minHCsats	0.00066
Smin34	0.000661
SHaaCH	0.000664
SIC3	0.000664
SHCsats	0.000681
Smin	0.000681
CrippenLogP	0.000682
maxsOH	0.000684
ATSc1	0.000684
bcutm13	0.000684
phi	0.000686
MATSm3	0.000688
CIC3	0.000688
VSAEstate7	0.000691
SPC-4	0.000695
EstateVSA7	0.000702
Smin8	0.000704
WTPT-5	0.000706
TPSA1	0.000708
naccr	0.00071
MATSm7	0.000712
maxdsN	0.000712
CIC1	0.000713
Smin35	0.000714
ATSe5	0.000716
minHCsatu	0.000725
GATSp3	0.000726
GATSm5	0.000727
ALogp2	0.000729
GATSp7	0.00073
EstateVSA1	0.000737
IDE	0.000741
mindO	0.000744
mChi1	0.000745
SaasC	0.00076
bcute9	0.000761
nAtomLAC	0.000762
maxdssC	0.000771
GATSe7	0.000775
Smax	0.000781
ETA_Epsilon_1	0.000787
MATSv5	0.000789
bcutp5	0.000793
IC1	0.000796
maxHBint7	0.000797
QCss	0.000823
CIC6	0.000823
ALogP	0.000826
bcutm3	0.00083
SsOH	0.000847
BertzCT	0.000851
EstateVSA4	0.000851
SdssC	0.000855
bcutm2	0.000866
MAXDN	0.000868
PC6	0.000872
MATSm6	0.000891
SHBint5	0.000897
SaaCH	0.0009
MATSp5	0.000901
MRVSA6	0.000904
slogPVSA1	0.000904
MATSm5	0.000922
bcute12	0.000926
J	0.000927
GATSm4	0.000927
MRVSA5	0.000933
MATSm1	0.000934
GATSm8	0.000939
Smin12	0.000946
hmin	0.00095
VC-4	0.000962
MATSe5	0.000963
MATSp4	0.000964
PEOEVSA5	0.000967
minHBd	0.000971
GATSv3	0.000974
bcutm9	0.000979
PEOEVSA8	0.00098
ECCEN	0.000987
MATSm8	0.000988
IC2	0.000995
BCUTp-1l	0.001004
minssCH2	0.001017
QHss	0.001019
Smax16	0.00102
bcutm12	0.001026
ETA_EtaP_F	0.001026
ETA_dEpsilon_D	0.001038
bcute4	0.001038
WTPT-3	0.001042
MAXDP2	0.001042
knotpv	0.001043
MDEO-11	0.001043
maxHCsats	0.00105
Chiv5ch	0.001063
GATSe5	0.001072
VPC-5	0.001081
MATSv8	0.00109
maxsF	0.001096
QNmin	0.001109
ETA_BetaP_s	0.001109
Chiv6ch	0.00111
IC3	0.001117
VPC-6	0.001119
VSAEstate2	0.001121
MATSp3	0.001137
slogPVSA2	0.00114
WTPT-4	0.001162
gmin	0.001163
minHBint6	0.001176
minHBint7	0.001195
Smax24	0.001225
MATSp6	0.001229
PEOEVSA1	0.001234
SIC2	0.001237
S34	0.001257
bcute1	0.001278
MATSv3	0.001281
SC-5	0.001283
dchi0	0.00129
SIC1	0.001291
maxHBd	0.001307
PEOEVSA7	0.001342
MDEC-24	0.001345
SCH-7	0.001347
SHBd	0.001349
MATSe8	0.001375
MATSv1	0.001375
SHCsatu	0.001386
Smin15	0.001398
BCUTp-1h	0.00141
GATSm3	0.001461
bcutp12	0.001465
MLFER_BH	0.001485
GATSv1	0.001559
QOmax	0.001589
slogPVSA0	0.001592
bcute10	0.001605
Smin24	0.001609
MATSp1	0.001616
Chiv3	0.001662
QNmax	0.001663
bcutv4	0.00168
VCH-5	0.001717
VSAEstate4	0.001785
ATSc5	0.001813
C3SP2	0.001831
mindssC	0.001846
ATSc2	0.001859
minHBint10	0.001866
ATSc3	0.001892
MDEC-22	0.001909
MAXDP	0.001935
knotp	0.001942
GATSm1	0.002
GATSp4	0.002026
maxsssCH	0.002031
S25	0.002032
bcutp1	0.002049
ETA_Shape_Y	0.002124
bcutp9	0.002186
XLogP	0.002237
ATSc4	0.002298
maxHBint5	0.002321
maxHBint8	0.002379
minsOH	0.002424
GATSm2	0.002443
SPC-6	0.00248
MATSe3	0.002549
MLFER_S	0.002597
SHBint6	0.002733
ndssC	0.002743
bcutv1	0.002787
VCH-7	0.002879
BCUTc-1l	0.002923
QCmax	0.00298
Scar	0.003191
minssO	0.003312
BCUTc-1h	0.003494
MLFER_A	0.003711
TopoPSA	0.003768
MDEO-12	0.003868
minHBa	0.004054
Smin33	0.004253
SHsOH	0.004402
GATSe8	0.004485
PEOEVSA6	0.00461
Mnc	0.004826
MATSe1	0.004978
LDI	0.005205
MDEC-33	0.005471
GATSe1	0.005843
bcute2	0.005866
VC-5	0.006197
nC	0.0064
nHBAcc	0.006408
LogP2	0.006781
SHBint10	0.006873
Hy	0.007517
kappam3	0.007695
VSAEstate1	0.007799
QNss	0.009891
minsssN	0.01014
LogP	0.011371
maxssO	0.011647
ATSp4.1	0.013044
QHmax	0.014923
C1SP2	0.01631
minHBint5	0.017225
ATSv5	0.017404
Smax35	0.018515
minHsOH	0.025883
maxHsOH	0.028849
LipoaffinityIndex	0.031403
QOmin	0.041317
Qmin	0.043254
MDEC-23	0.049635
ATSp5.1	0.143226

The article "Optimization Method of an Antibreast Cancer Drug Candidate Based on Machine Learning" was published in 2022. Journal: Comput Math Methods Med.

**Table 2:** Quantitative prediction accuracy of biological activity.

Biological activity	MSE	MAPE	MAE
pIC50	1.5720	0.1624	0.9880

**Table 3:** Qualitative prediction accuracy of biological activity.

ADMET	Accuracy	Precision	Recall	F1 score
Caco-2	0.8830	0.8158	0.3735	0.5124
CYP3A4	0.8230	0.8286	0.7436	0.7838
hERG	0.7660	0.7091	0.5147	0.6142
HOB	0.7979	0.5263	0.1333	0.2127
MN	0.9149	0.9444	0.7907	0.8608

**Table 4:** The predicted values for best-performance candidate's operating variables.

Descriptor	Normalized	Real
ALogP	0.796372	22.52675
ALogp2	0.565526	301.9008
nC	0.911078	80.17483
ATSc1	0.49451	2.244443
ATSc2	0.939863	2.221841
ATSc3	0.15546	0.141572
ATSc4	0.452555	1.233483
ATSc5	0.454323	1.587603
BCUTc-1l	0.086871	0.020243
BCUTc-1h	0.197627	0.09002
BCUTp-1l	0.348526	1.416559
BCUTp-1h	0.30613	2.687486
C1SP2	0.842156	16.84312
C3SP2	0.44475	5.337003
SCH-7	0.570198	1.226224
VCH-5	0.136673	0.066583
VCH-7	0.284164	0.471843
SC-5	0.90026	2.358201
VC-4	0.678221	0.33911
VC-5	0.476908	0.706329
SPC-4	0.223485	4.435693
SPC-6	0.734395	25.70635
VPC-5	0.126582	1.515056
VPC-6	0.017549	0.319702
CrippenLogP	0.908239	23.01173
ECCEN	0.868879	13130.5
ndssC	0.095972	2.687217
SHBd	0.814323	14.78969
SHBint5	0.536753	51.89493
SHBint6	0.493409	88.24471
SHBint10	0.622465	71.61779
SHsOH	0.680758	1.868451
SHaaCH	0.943556	9.03814
SHCsats	0.361675	16.73021
SHCsatu	0.005772	0.112306
SaaCH	0.522805	20.98883
SdssC	0.131028	4.567775
SaasC	0.472381	10.71859
SsOH	0.945776	62.06689
minHBd	0.004693	0.004157
minHBa	0.381193	6.144505
minHBint5	0.414706	5.288915
minHBint6	0.647892	5.650089
minHBint7	0.123079	1.481101
minHBint10	0.785248	9.487377
minHsOH	0.825143	0.730969
minHCsats	0.59855	0.663469
minHCsatu	0.105526	0.118007
minssCH2	0.889895	2.358533
mindssC	0.268325	1.054303
minsssN	0.735504	2.011435
minsOH	0.967622	11.35247
mindO	0.231127	3.32619
minssO	0.222965	1.499747
maxHBd	0.573001	0.488639
maxHBint5	0.502949	5.811736
maxHBint7	0.117421	1.2678
maxHBint8	0.185541	1.72333
maxHsOH	0.609498	0.519763
maxHCsats	0.973025	1.252399
maxsssCH	0.255134	0.249398
maxdssC	0.322333	0.754448
maxdsN	0.148611	0.763495
maxsOH	0.982069	12.24723
maxssO	0.754777	5.077492
maxsF	0.375781	5.816332
hmin	0.202651	0.19802
gmin	0.196719	1.518661
LipoaffinityIndex	0.351299	9.693234
MAXDN	0.916639	5.952869
MAXDP	0.688238	4.738658
MAXDP2	0.41876	2.882345
ETA_Epsilon_1	0.744645	0.275913
ETA_dEpsilon_D	0.389612	0.062396
ETA_Shape_Y	0.912192	0.399887
ETA_BetaP_s	0.60827	0.118229
ETA_EtaP_F	0.156509	0.243636
nHBAcc	0.763162	50.36871
nAtomLAC	0.886048	15.94887
MDEC-14	0.861766	4.024826
MDEC-22	0.385049	13.60019
MDEC-23	0.253417	13.6896
MDEC-24	0.187219	2.285725
MDEC-33	0.722608	35.96141
MDEO-11	0.339665	1.592459
MDEO-12	0.690197	2.438236
MLFER_A	0.884812	7.618233
MLFER_BH	0.682306	15.75445
MLFER_S	0.983677	20.57753
TopoPSA	0.810281	968.5693
WTPT-3	0.939527	169.2643
WTPT-4	0.836226	42.47587
WTPT-5	0.580833	73.03263
XLogP	0.921274	16.46778
kappam3	0.591715	38.51945
phi	0.069879	4.911113
LDI	0.839175	0.266858
Mnc	0.401081	0.122731
QNss	0.717554	3.800167
QCss	0.401335	0.675045
QHss	0.816212	1.412047
Qmin	0.458487	0.197608
QOmin	0.902885	0.557983
QNmin	0.399317	0.186082
QOmax	0.2189	0.111201
QNmax	0.733215	0.462658
QCmax	0.219663	0.114005
QHmax	0.309301	0.08877
mChi1	0.70787	0.059461
knotp	0.463493	3.682452
Chiv3	0.504351	12.68139
dchi0	0.531787	14.54385
Chiv5ch	0.373625	0.159538
Chiv6ch	0.813352	0.252139
knotpv	0.332321	1.601785
naccr	0.252895	8.092637
PC6	0.68057	207.574
S17	0.617016	13.29916
S25	0.41233	3.873014
S34	0.471534	30.94445
Smax11	0.012002	0.028529
Smax16	0.270107	0.819234
Smax24	0.166683	0.618393
Smax35	0.118755	0.798862
Smin8	0.95032	2.519298
Smin12	0.345704	1.386271
Smin15	0.094406	0.351002
Smin24	0.795928	2.952893
Smin33	0.561019	6.58187
Smin34	0.555043	7.947103
Smin35	0.727286	4.891723
Scar	0.881448	89.12223
Smax	0.089706	1.067416
Smin	0.953752	6.591381
GATSm1	0.812402	1.001692
GATSm2	0.634299	0.793508
GATSm3	0.120694	0.223285
GATSm4	0.510951	0.973362
GATSm5	0.049626	0.135925
GATSm8	0.100571	0.559475
GATSv1	0.961747	0.951168
GATSv3	0.282006	0.472642
GATSe1	0.927808	0.905541
GATSe5	0.599223	1.181668
GATSe7	0.23859	1.199867
GATSe8	0.078374	0.43999
GATSp3	0.437899	0.708521
GATSp4	0.924518	1.591095
GATSp7	0.980757	4.932225
TPSA1	0.606654	694.4674
slogPVSA0	0.062831	13.0085
slogPVSA1	0.216952	76.48269
slogPVSA2	0.700064	67.12981
MRVSA5	0.64033	57.65721
MRVSA6	0.374169	51.50251
PEOEVSA1	0.302775	42.13574
PEOEVSA5	0.643223	105.9755
PEOEVSA6	0.965518	159.7043
PEOEVSA7	0.010657	0.809047
PEOEVSA8	0.929568	51.26194
EstateVSA1	0.420173	90.7544
EstateVSA4	0.150524	17.979
EstateVSA7	0.617028	85.38316
VSAEstate1	0.916056	260.2258
VSAEstate2	0.469295	61.3763
VSAEstate4	0.182115	5.816037
VSAEstate7	0.434015	9.820449
MATSm1	0.259205	0.199588
MATSm3	0.55142	0.600496
MATSm5	0.41914	0.43381
MATSm6	0.11384	0.224834
MATSm7	0.309463	0.536608
MATSm8	0.835615	8.049475
MATSv1	0.691362	0.486719
MATSv3	0.421519	0.464936
MATSv5	0.803173	1.224839
MATSv8	0.974739	10.77086
MATSe1	0.044383	0.029914
MATSe3	0.858027	0.967855
MATSe5	0.820808	0.897964
MATSe8	0.84285	8.119175
MATSp1	0.618676	0.638474
MATSp3	0.031658	0.035141
MATSp4	0.995234	1.393328
MATSp5	0.310054	0.464771
MATSp6	0.950285	1.76563
MATSp7	0.401141	0.920218
ATSv5	0.422807	1.369895
ATSe5	0.526873	1.836152
ATSp4.1	0.970895	2.954435
ATSp5.1	0.441556	1.408123
J	0.517201	2.905116
BertzCT	0.331505	0.429631
IDE	0.017944	0.054297
LogP	0.809566	20.63664
LogP2	0.935064	170.3864
Hy	0.258499	0.832883
CIC1	0.531694	2.274054
CIC3	0.195279	0.597359
CIC4	0.947302	2.624027
CIC6	0.315254	0.833533
SIC1	0.534191	0.238783
SIC2	0.548336	0.223173
SIC3	0.93592	0.379048
IC1	0.62343	1.283018
IC2	0.961285	2.260943
IC3	0.605757	1.788194
bcutm13	0.686797	0.80836
bcutm12	0.096662	0.106618
bcutm9	0.662882	0.380495
bcutm3	0.045307	0.169084
bcutm2	0.449717	3.285183
bcutv4	0.772798	0.863988
bcutv1	0.57612	0.338759
bcute12	0.330634	0.366674
bcute10	0.721806	0.510317
bcute9	0.529904	0.349736
bcute4	0.370874	0.411299
bcute2	0.741989	0.470421
bcute1	0.128208	0.061027
bcutp12	0.873497	0.828075
bcutp9	0.541204	0.357195
bcutp5	0.669777	0.953092
bcutp1	0.884249	0.579183

The article "Optimization Method of an Antibreast Cancer Drug Candidate Based on Machine Learning" was published in 2022. Journal: Comput Math Methods Med.

## Data Availability

The datasets used during the current study are available from the corresponding author upon reasonable request.
